# Timing Decision of Low-Carbon Technology Investment Adoption by High Energy Consuming Enterprises under Carbon Trading and Subsidies

**DOI:** 10.1155/2022/9848994

**Published:** 2022-11-17

**Authors:** Bin Li

**Affiliations:** College of Economics & Management, Taiyuan University of Technology, Shanxi 030002, China

## Abstract

Although government subsidies provide some financial support for firms to invest in low-carbon technologies, carbon price fluctuations bring greater uncertainty risks to firms' investment. The paper constructs a real option model to analyze the timing of low-carbon technology adoption between upstream dominant high energy consuming firms and downstream retailers in case of collaborative decision-making and Stackelberg game, and a numerical simulation is conducted to analyze factors affecting the timing for low-carbon investment. We find that the proportion of cost subsidies, carbon price volatility, carbon emission reduction rate, and cost-sharing ratio will affect firms to choose the optimal investment opportunity.

## 1. Introduction

High energy consuming enterprises have become the main carbon emission units. Because they consume more fossil energy, they bring higher carbon emissions, but have higher emission reduction potential and efficiency. The innovation and adoption of low-carbon technology by high energy consuming enterprises is an important way to achieve China's “carbon peaking and carbon neutrality” goal, and the carbon emission trading market established in China can have an impact and can promote enterprises to adopt low-carbon technology through the role of market mechanism. In recent years, China's carbon price fluctuates frequently, which brings great uncertainty risk to enterprises' low-carbon technology investment, and enterprises will wait to find the best investment opportunity. At the same time, the government has issued a series of subsidies and preferential policies to mobilize the enthusiasm of high energy consuming enterprises to invest in low-carbon technologies and accelerate the investment process of enterprises. Therefore, it is of great significance to evaluate the risks and investment opportunities of low-carbon technology adoption by high energy consuming enterprises under carbon trading and government subsidy policies.

The concept of low-carbon development has permeated all walks of life. Many scholars have studied the management of carbon emissions and the decision-making of emission reduction in different industries and fields. Bi et al. built an incentive mechanism based on a unified queueing, neural network model to enhance the energy efficiency of the urban transportation network [1]. Liu et al. has built an integer scheduling model to optimize the transportation path for the problem of high energy consumption in the field of cold chain fresh logistics [2]. Liu et al. discussed the low-carbon decision-making of automotive parts supply chain based on the smart city construction context [3]. In order to improve the robustness of urban road network and energy efficiency, Shang et al. analyze the topological characteristics of urban road network, a new method for measuring the robustness of road interruption was proposed [4, 5]. With the introduction of complex network, Shang et al. has discussed the impact of COVID-19 pandemic on user behavior and environmental benefits of shared bicycles through big data [6]. Most of the existing literature examines the impact of carbon trading and carbon taxes on carbon reduction investments from the perspective of government policy. Richstein et al. developed carbon price difference (ccfds) contracts to reduce the risk of investment in political and market uncertainty given the higher operating and investment costs faced by low-carbon investment in the steel industry and the insufficient and uncertain carbon price [7]. Hasan et al. exemplify warehouse operation and transportation logistics system as emission sources, and develop three models to optimize carbon tax, quota and transaction, inventory level, and technology investment decision under strict regulations on carbon restrictions [8]. Liu et al. investigated the impact of government regulation policies on the stabilization strategy of reducing emissions in the supply chain of green products and medical recycling by building an evolutionary game model [9, 10]. Yan et al. took power companies as an example to discuss the impact of different strategic combinations of carbon quota and trading mechanism, the standard policy of renewable energy portfolio [11]. Lu et al., taking carbon cap trading and carbon offset policy into account, constructed a Stackelberg game model, studied the optimal solution between supplier and buyer, and analyzed its influencing factors [12]. Zhang et al., taking iron and steel companies as an example, an evolutionary game model is constructed to discuss the strategic choice between large and medium enterprises under government subsidy and carbon trading mechanism [13]. Comparison of different emission reduction strategies by Liu et al. found it difficult to achieve the coordination of supply chain benefits by relying solely on carbon taxation policies [14]. Yi et al. considered consumers' low-carbon preferences and considered the effect of green subsidies and emission taxes on improving green innovation in the supply chain consisting of producers and retailers [15]. Bai et al. established two optimization models of technology investment with and without manufacturer-led guidance and studied the impact of contribution in maintainability innovation on supply chain finance and natural execution [16]. Taking OECD countries as an example, Ganda et al. researched on the role of investments in innovation and technology in improving environmental quality [17]. Liu et al. focused on agricultural carbon emissions and discussed the impact of carbon taxes and investment cooperation on decisions to reduce emissions from agricultural supply chains through game modeling [18]. Some researchers have also used the real options model to study investment decision-making in carbon emission reduction. Liu et al., to evaluate the investment value and timing based on the impact of innovation learning, developed a new model of real option investment decision-making and proposed a two-figure component-based innovation learning curve method to anticipate the end of the toll taken on each component [19]. Compernolle et al. built a dynamic real options model to analyze the impact of positively correlated price uncertainty on the decision time of investment [20].

Most existing studies have investigated supply chain coordination and investment decision-making in carbon emission reduction from the perspective of carbon trading, carbon taxes, and consumer preference for low-carbon emissions. Few studies, however, have investigated the timing of low-carbon technology investment in both scenarios of collaborative decision-making and Stackelberg game from the perspective of carbon trading and the government subsidy composite politics. Thus, this paper studies the decision-making of low-carbon technology investment of high energy consuming enterprises under the dual carbon trading and government subsidy policies, solves the enterprise investment threshold driven by government policies, and analyzes the impact of carbon price fluctuations and the proportion of government subsidies on the timing of low-carbon technology investment, so as to provide a basis for low-carbon investment of enterprises and to provide the government with a reference for formulating a more focused whole.

## 2. Problem Description and Basic Assumptions

**Hypothesis 1 .**

High energy consuming enterprises only make one product, and the product sales volume reaches the annual maximum production capacity of the enterprise is *Q* (constant). The adoption of low-carbon technology has no impact on production efficiency, this investment is irreversible, and the enterprise's risk appetite is neutral. After adopting low-carbon technology, high energy consuming enterprises will immediately obtain carbon emission reduction amount and hold it for a long time and can invest at the earliest at moment *t* = 0.

**Hypothesis 2 .**

Suppose that the carbon emission per unit item before the adoption of low-carbon technology is *e*_0_, the carbon emission per unit product after the adoption of low-carbon technology is *e*, the emission reduction rate of low-carbon technology is *η* = *e*_0_ − *e*/*e*_0_, and the one-time investment cost of carbon emission reduction technology for high energy consuming enterprises is 1/2*λη*^2^, of which *λ* is the cost coefficient of high energy consuming enterprises adopting low-carbon technology and on behalf of the cost level of low-carbon technology.

**Hypothesis 3 .**

Suppose that the price of carbon emission right at time *t* is *p*_*c*_(*t*), and it obeys geometric Brownian motion, which satisfies

(1) $$\begin{array}{c} d_{p_{c}\left(t\right)}=\alpha p_{c}\left(t\right)\text{dt}+\beta p_{c}\left(t\right)d_{z\left(t\right)}. \end{array}$$

Among them, *α* > 0 and *β* > 0 are the drift term and variance, the drift coefficient is the expected growth rate, and meets 0 ≤ *α* < *r* (*r* is the risk-free interest rate, which is measured by the average return rate of the capital market), and *β* the variance represents the carbon price fluctuation; *d*_*z*(*t*)_ is the increment of the standard Wiener process, and there is *d*_*z*(*t*)_ ~ *N*(0, *d*_*t*_) [21]; *dt* is the time interval of infinite approaching zero.

**Hypothesis 4 .**

The government gives a certain cost subsidy to high energy consuming enterprises for low-carbon technology investment, and the subsidy proportion is *μ*.

## 3. Model Construction and Optimal Adoption Timing Analysis

### 3.1. Collaborative Decision Analysis

#### 3.1.1. Model Building

Suppose that high energy consuming enterprises adopt low-carbon technology at time *t*, and the adoption of low-carbon technology is an investment that can benefit for a long time. Considering that the random fluctuation of carbon commerce value can manufacture uncertainty risk, real choices are often wont to evaluate the expectation of carbon emission reductions within the carbon commerce market. The expected net income of enterprises after adopting emission reduction technology is

(2) $$\begin{array}{c} W\left(t\right)=E\left[\int_{t}^{\infty }p\left(s\right)\eta e_{0}{Qe}^{-r\left(s-t\right)}\text{ds}-\frac{1-\mu }{2}{\lambda \eta }^{2}\right]=\frac{\eta e_{0}Qp\left(t\right)}{r-\alpha }-\frac{1-\mu }{2}{\lambda \eta }^{2}. \end{array}$$

#### 3.1.2. Analysis of Emission Reduction Technology Adoption Threshold

The risk attitude of the enterprise is risk neutral. Therefore, the adoption of emission reduction technology will be considered only when it is profitable; that is, when the expected investment income of high energy consuming enterprises adopting emission reduction technology is positive, then Equation (2) must be satisfied that is greater than or equal to 0; that is, when *p*(*t*) ≥ (1 − *μ*)(*r* − *α*)*λη*/2*e*_0_*Q*, it is profitable for high energy consuming enterprises to invest in emission reduction technology, so that *p*^∗^ is the threshold carbon price for high energy consuming enterprises to adopt emission reduction technology, then

(3) $$\begin{array}{c} p^{*}=\frac{\left(1-\mu \right)\left(r-\alpha \right)\lambda \eta }{2e_{0}Q}. \end{array}$$

#### 3.1.3. Analysis of Investment Opportunity of Low-Carbon Technology

Before adopting low-carbon technologies, high energy consuming enterprises hold investment options and do not generate carbon trading gains during the waiting period. High energy consuming enterprises will choose the time of adoption according to the principle of maximizing the expected return of the adoption of low-carbon technologies; that is, they will stop waiting for the implementation of investment actions until the trading price of carbon emission rights reaches the adoption threshold for the first time at a certain time. Therefore, this problem is an optimal stopping time problem.

Before adopting low-carbon technology, for supply chain enterprises, the adoption opportunity of low-carbon technology can be regarded as a real option equity owned by them, which is determined by the change profit and loss of option value of carbon emission reduction obtained by adopting low-carbon technology. In the waiting range, the change of option value satisfies Bellman equation:rWdt = *E*[dW].

Combined with Ito lemma, the expected value function of call option satisfies the differential equation: (1/2)*β*^2^*p*^2^*W*^″^ + (*r* − *α*)*pW*′ − *rW* = 0.

The general solution of the above formula is *W* = *C*_1_*p*^*ζ*_1_^ + *C*_2_*p*^*ζ*_2_^, where *ζ*_1_ and *ζ*_2_ are constants.

It can be deduced from the conclusion of Dixit and pingdyck: *C*_2_ = 0,$\zeta_{1}=\left(1/2\right)-\left(\alpha /\beta^{2}\right)+\sqrt{{\left(\left(\alpha /\beta^{2}\right)-\left(1/2\right)\right)}^{2}+2r/\beta^{2}}>1$.

Assuming that high energy consuming enterprises stop waiting for investment actions at time *T*, the expected benefits of adopting low-carbon technologies can be maximized. Let *W*_*T*_ represents the option value function of the income from emission reduction technology adoption, then

(4) $$\begin{array}{c} W_{T}=\underset{T\geq 0}{\max}E\left[\left(\frac{\eta e_{0}Qp\left(t\right)}{i-\mu }-\frac{1-\mu }{2}{\lambda \eta }^{2}\right)e^{-r\left(t-T\right)}\right]. \end{array}$$

From *E*[(*ηe*_0_*Qp*(*t*)/*r* − *α*) − (1 − *μ*/2)*λη*^2^]*e*^−*r*(*t* − *T*)^ = ((*ηe*_0_*Qp*_*T*_/*r* − *α*) − (1 − *μ*/2)*λη*^2^)(*p*(*t*)/*p*_*T*_)^*ζ*^,order (*∂*/*∂p*_*T*_)((*ηe*_0_*Qp*_*T*_/*r* − *α*) − (1 − *μ*/2)*λη*^2^)(*p*(*t*)/*p*_*T*_)^*ζ*^ = 0, and the optimal adopted carbon price of emission reduction technology is

(5) $$\begin{array}{c} p_{T}^{**}=\frac{\zeta }{\zeta -1}\frac{\left(1-\mu \right)\lambda \eta }{2e_{0}Q}\left(r-\alpha \right). \end{array}$$

By observing Equations (3) and (5), it can be found that the optimal adopted carbon price *p*_*T*_^∗∗^ is more than the threshold carbon price *p*^∗^ by a factor of (*ζ*/*ζ* − 1) > 1, indicating that the threshold carbon price is the carbon price level at the breakeven point of adopting emission reduction technology, and the carbon price level of the best investment opportunity of supply chain enterprises is higher than the threshold carbon price.

Inference 1: the threshold carbon price of emission reduction technology *p*_*T*_^∗∗^ is in direct proportion to the carbon emission reduction rate *η*, and increases with the increase of carbon emission reduction rate *η*, indicating that with the increase of carbon emission reduction rate, the threshold carbon price of high- and low-carbon technology adoption will be pushed, delaying the adoption of emission reduction technology. On the contrary, the lower the carbon emission reduction rate is, the lower the threshold carbon price will be. Supply chain enterprises choose to adopt emission reduction technologies, which can speed up the adoption process.

Inference 2: the threshold carbon price *p*_*T*_^∗∗^ is inversely proportional to the cost subsidy ratio *μ*, and decreases with the increase of the cost subsidy ratio *μ*, indicating that if the government increases the cost subsidy ratio, it will reduce the investment threshold for supply chain enterprises to adopt emission reduction technologies and accelerate the process of emission reduction technology adoption. When the proportion of government cost subsidies is high, it eases some of the financial pressure on enterprises, and is conducive to enhancing the willingness of enterprises to adopt low-carbon technologies, thereby accelerating the adoption process. When the proportion of cost subsidies is low, emission reduction technology investment is difficult to receive returns in the short term, and requires more funds. Therefore, enterprises will delay investment and wait for the opportunity for higher returns from the adoption of emission reduction technologies.

In the case of collaborative decision-making, the option value *W* of the supply chain adopting emission reduction technology can be expressed as

(6) $$\begin{array}{c} W\left(p\left(t\right)\right)=\left\{\begin{array}{c} \left(\frac{\eta e_{0}{Qp}_{T}^{**}}{r-\alpha }-\frac{1-\mu }{2}{\lambda \eta }^{2}\right){\left(\frac{p\left(t\right)}{p_{T}^{**}}\right)}^{\lambda },p\left(t\right)<p_{T}^{**}\\ \frac{\eta e_{0}{Qp}_{T}^{**}}{r-\alpha }-\frac{1-\mu }{2}{\lambda \eta }^{2},p\left(t\right)\geq p_{T}^{**} \end{array}\right.. \end{array}$$

The corresponding optimal investment opportunity is

(7) $$\begin{array}{c} T^{*}=\frac{\ln\left(p_{T}^{**}/p_{c0}\right)}{\alpha -\left(\beta^{2}/2\right)}=\frac{\ln\left(\left(\zeta /\zeta -1\right)\left[\left(\left(1-\mu \right)\lambda \eta /2e_{0}Q\right)-k\right]\left(r-\alpha \right)/p_{c0}\right)}{\alpha -\left(\beta^{2}/2\right)}, \end{array}$$

_where_*T*^∗^_is the moment when the carbon price reaches the optimal investment threshold for the first time._

### 3.2. Stackelberg Game Analysis

#### 3.2.1. Stackelberg Game Model

Based on the basic supply chain model, this paper further analyzes the investment opportunity of emission reduction technology under the scenario of cooperation between enterprises within the supply chain. Assuming that in the supply chain, high energy consuming enterprises are the leaders in adopting emission reduction technologies, and the proportion of emission reduction technology projects requiring retailers to jointly bear the total cost of adoption investment is *θ* (0 ≤ *θ* ≤ 1), the investment amount of retailers is *θI*, and the investment amount of high energy consuming enterprises is (1 − *θ*)*I*. If the high energy consuming enterprise promises to pay the carbon trading market income to the retailer in proportion of *γ* (0 ≤ *γ* ≤ 1), the present value of the net investment income of the high energy consuming enterprise adopting low-carbon technology is

(8) $$\begin{array}{c} W_{M}\left(t\right)=E\left\{\int_{t}^{\infty }\left[p\left(s\right)\eta e_{0}Q\left(1-\gamma \right)\right]e^{-r\left(s-t\right)}ds\right\}-\frac{1-\mu }{2}{\lambda \eta }^{2}\left(1-\theta \right)=\frac{\eta e_{0}Qp\left(t\right)}{r-\alpha }\left(1-\gamma \right)-\frac{1-\mu }{2}{\lambda \eta }^{2}\left(1-\theta \right). \end{array}$$

The present value of the expected net income of retailers' investment in adopting low-carbon technology is

(9) $$\begin{array}{c} W_{R}\left(t\right)=E\left\{\int_{t}^{\infty }\left[p\left(s\right)\eta e_{0}Q\gamma \right]e^{-r\left(s-t\right)}ds\right\}-\frac{1}{2}{\theta \lambda \eta }^{2}=\frac{\eta \gamma e_{0}Qp\left(t\right)}{r-\alpha }-\frac{1}{2}{\theta \lambda \eta }^{2}. \end{array}$$

When solving the problem, we can first find out the time when retailers adopt low-carbon technology according to the expected net income function, then deduce the transfer payment proportion of high energy consuming enterprises, and finally obtain the time of supply chain technology investment.

Use Ito lemma and Bellman equation to solve the optimal investment opportunity of retailers.

The value function of retailers waiting for the adoption of low-carbon technologies is

(10) $$\begin{array}{c} W_{R}\left(T\right)=\underset{T\geq 0}{\max}E\left[\left(\frac{\eta \gamma e_{0}Qp\left(t\right)}{r-\alpha }-\frac{1-\mu }{2}{\theta \lambda \eta }^{2}\right)e^{-r\left(t-T\right)}\right]. \end{array}$$

From *E*[((*ηγe*_0_*Qp*(*t*)/*r* − *α*) − (1 − *μ*/2)*θλη*^2^)*e*^−*r*(*t* − *T*)^] = ((*ηγe*_0_*Qp*_*T*_/*r* − *α*) − (1 − *μ*/2)*θλη*^2^)(*p*(*t*)/*p*_*T*_)^*ζ*^,order (*∂*/*∂p*_*T*_)((*ηγe*_0_*Qp*_*T*_/*r* − *α*) − (1 − *μ*/2)*θλη*^2^)(*p*(*t*)/*p*_*T*_)^*ζ*^ = 0, the best adopted carbon price of low-carbon technology available to retailers is

(11) $$\begin{array}{c} p_{\text{TR}}=\frac{\zeta }{\zeta -1}\frac{\theta \lambda \eta }{2\gamma e_{0}Q}\left(r-\alpha \right)\left(1-\mu \right). \end{array}$$

At this time, the optimal investment opportunity for retailers is

(12) $$\begin{array}{c} T_{R}^{**}=\frac{\ln\left(p_{\text{TR}}/p_{c0}\right)}{\alpha -\left(\beta^{2}/2\right)}=\frac{\ln\left(\left(\zeta /\zeta -1\right)\left(\theta \lambda \eta /2\gamma e_{0}Q\right)\left(r-\alpha \right)\left(1-\mu \right)\right)}{\alpha -\left(\beta^{2}/2\right)}. \end{array}$$

The option value of retailers' investment in low-carbon technology is

(13) $$\begin{array}{c} W_{R}\left(p\left(t\right)\right)=\left\{\begin{array}{c} \left(\frac{\eta \gamma e_{0}{Qp}_{\text{TR}}}{r-\alpha }-\frac{1-\mu }{2}{\theta \lambda \eta }^{2}\right){\left(\frac{p\left(t\right)}{p_{\text{TR}}}\right)}^{\zeta },p\left(t\right)<p_{\text{TR}}\\ \frac{\eta \gamma e_{0}{Qp}_{\text{TR}}}{r-\alpha }-\frac{1-\mu }{2}{\theta \lambda \eta }^{2},p\left(t\right)\geq p_{\text{TR}} \end{array}\right.. \end{array}$$

Inference 3: In the Stackelberg game, the retailer's optimal adopted carbon price *p*_TR_ and the optimal investment opportunity *T*_*R*_^∗∗^ are inversely proportional to the cost subsidy ratio *θ*; that is, the higher the subsidy ratio given by the government, the lower the retailer's optimal adopted carbon price for adopting low-carbon technology, and the adoption will be implemented in advance. On the contrary, the lower the subsidy proportion given by the government, the higher the optimal adoption carbon price of retailers will be, and the adoption of low-carbon technologies will be postponed.

Inference 4: In the Stackelberg game, the retailer's optimal adoption of carbon price *p*_TR_ and the optimal investment opportunity *T*_*R*_^∗∗^ are proportional to the proportion of cost sharing *θ*; that is, the higher the proportion of investment cost shared by the retailer, the higher the retailer's optimal adoption of carbon price, which will delay the adoption of emission reduction technology. On the contrary, the lower the proportion of investment cost shared by retailers, the lower the optimal adopted carbon price of retailers will be, and the optimal investment opportunity will be advanced.

#### 3.2.2. Analysis on the Transfer Payment Proportion of Carbon Trading Income of High Energy Consuming Enterprises

After deriving the optimal investment threshold and expected return of retailers, high energy consuming enterprises should determine the transfer payment proportion *γ* according to the timing of retailers' adoption of emission reduction technology to ensure the maximization of their expected return.

The option value function of the manufacturer during the waiting period for the adoption of emission reduction technology is

(14) $$\begin{array}{c} W_{M}\left(p\left(t\right)\right)=\left[\frac{\eta e_{0}{Qp}_{\text{TR}}}{r-\alpha }\left(1-\gamma \right)-\frac{1-\mu }{2}{\lambda \eta }^{2}\left(1-\theta \right)\right]{\left(\frac{p\left(t\right)}{p_{\text{TR}}}\right)}^{\zeta }. \end{array}$$

Find the first derivative of the above formula for *γ* and make it 0 to obtain

(15) $$\begin{array}{c} \gamma_{1}=\frac{\theta \zeta -\theta }{\theta +\zeta -1}. \end{array}$$

And considering the boundary condition (*ηγe*_0_*Qp*_0_/*i* − *μ*) − (1/2)*θβη*^2^ ≥ 0 that the retailer's income needs to meet, we get

(16) $$\begin{array}{c} \gamma_{2}=\frac{\theta \beta \eta \left(i-\mu \right)}{2e_{0}{Qp}_{0}}. \end{array}$$

Then, the optimal transfer payment proportion of carbon trading income that high energy consuming enterprises can choose is

(17) $$\begin{array}{c} \gamma =\min\left\{\frac{\theta \zeta -\theta }{\theta +\zeta -1},\frac{\theta \beta \eta \left(i-\mu \right)}{2e_{0}{Qp}_{0}}\right\}. \end{array}$$

#### 3.2.3. Timing of Supply Chain Adoption

In the Stackelberg game, the overall expected return of the supply chain is *W*_*S*_ = *W*_*M*_ + *W*_*R*_. Referring to the collaborative decision-making derivation process, it can be concluded that the optimal carbon price for the adoption of emission reduction technology in the supply chain is

(18) $$\begin{array}{c} p_{T}^{***}=\frac{\zeta \lambda \eta \left(1-\mu \right)}{2e_{0}Q\left(\zeta ‐1\right)}\left(1+\frac{\theta }{\zeta -1}\right). \end{array}$$

The optimal investment opportunity in the Stackelberg game is obtained as follows:

(19) $$\begin{array}{c} T^{***}=\frac{\ln\left(p_{T}^{***}/p_{c0}\right)}{\alpha -\left(\beta^{2}/2\right)}=\frac{\ln\left(\left(\zeta \lambda \eta \left(1-\mu \right)/2e_{0}Q\left(\zeta ‐1\right)\right)\left(1+\left(\theta /\zeta -1\right)\right)\right)}{\alpha -\left(\beta^{2}/2\right)}. \end{array}$$

## 4. Simulation Analysis

### 4.1. Collaborative Decision Analysis

Assign parameters to the low-carbon technology adoption decision-making model: *α* = 0.05, *r* = 0.8, *e*_0_ = 5, *λ* = 500000, *Q* = 1000, and*β* value separately 0.3, 0.6, and 0.9.

From Figure 1, the optimal adopted carbon price increases with the increase of carbon emission reduction rate; that is, the greater the carbon emission reduction rate, the higher the optimal adopted carbon price. With the reduction of enterprise carbon emissions, enterprises can sell more excess carbon emissions and obtain more benefits from the carbon trading market. Therefore, enterprises will delay the adoption of low-carbon technologies and wait for higher opportunities for carbon trading benefits, which verifies inference 1. In addition, the optimal adoption of carbon price increases with the increase of carbon price volatility. The greater the fluctuation of carbon price, the higher the risk of carbon trading. Enterprises will delay the adoption of low-carbon technologies and wait for better investment opportunities.

From Figure 2, the optimal adopted carbon price decreases with the rise of the proportion of value subsidies; that is, the higher the proportion of cost subsidies, the lower the optimal adopted carbon price of enterprises under collaborative decision-making, which indicates that when the government increases the proportion of cost subsidies, enterprises will accelerate the adoption of emission reduction technologies to reduce carbon emissions, which verifies inference 2.

### 4.2. Stackelberg Game Decision Analysis

Assign parameters to the low-carbon technology adoption decision-making model: *α* = 0.05, *r* = 0.8, *e*_0_ = 5, *λ* = 500000, *Q* = 1000, *η* = 0.5, *γ* = 0.5, and *β* value separately 0.3, 0.6, and 0.9.

1. It can be seen from Figure 3 that the value of optimal use of carbon decreases with the increase of the value subsidy proportion; that is, the upper the proportion of subsidies given by the govt. to high energy intense enterprises, the lower the optimum adoption carbon value of low-carbon technology by retailers, which is able to promote them to participate within the cooperation of adopting emission reduction technology within the provide chain prior to, that verifies inference 3
2. As shown in Figure 3, the optimal adopted carbon price increases with the increase of the cost sharing ratio; that is, the more the retailer shares the cost, the higher the optimal adopted carbon price level. At this time, the retailer will delay the opportunity to participate in the supply chain to adopt emission reduction technology and wait for a better investment opportunity, which verifies inference 4

From Figure 4, it can be seen that the proportion of transfer payment is inversely proportional to the optimal carbon price adopted by retailers, and the larger the proportion of carbon trading income given by high energy consuming enterprises to retailers, the lower the optimal carbon price adopted, and retailers will choose to invest in emission reduction technologies in advance.

## 5. Conclusion

High energy consuming enterprises need to purchase carbon emission rights in the carbon trading market in order to meet the government's environmental protection standards due to their large carbon emissions, so they are more vulnerable to the impact of carbon trading price fluctuations. Under the compound policy of carbon trading and government subsidies, carbon trading prices fluctuate frequently, making high energy consuming enterprises face greater uncertainty risks when investing in low carbon technologies, and government subsidies provide some support for high energy consuming enterprises to adopt low-carbon technologies. This paper analyzes the impact of carbon price fluctuations and government subsidies on the optimal timing of low-carbon technology investment of high energy consuming enterprises by constructing a real option model.

The main conclusions are as follows: (1) In the case of cooperative decision-making, the greater the fluctuation in carbon trading value, the higher the uncertainty risk presented by firms, and consequently, intense high-energy firms delay low-carbon investment; once the government increases the proportion of subsidies, it will relieve the monetary pressure on the offer chain firms and accelerate investment in low-carbon technologies.

(2) In the Stackelberg game, increasing the proportion of government subsidies will speed up the process of retailers adopting low-carbon technologies, but the higher the proportion that retailers share costs, the more likely they are to delay investing in low-carbon technology

This paper investigates the impact of carbon trading and government subsidy policies on the timing of low-carbon investment by companies. In the actual investment process, however, firms will also be affected by factors such as consumers' low-carbon preference and firms' investment risk attitude. This is also the direction of future research.

## Figures and Tables

**Figure 1:** Impact of carbon emission rate on optimal adopted carbon price.

**Figure 2:** Impact of cost subsidy proportion on the optimal adopted carbon price.

**Figure 3:** Impact of cost subsidy proportion and cost sharing ratio on retailers' optimal adopted carbon price.

**Figure 4:** Impact of transfer payment ratio on retailers' optimal adoption of carbon price.

## Data Availability

The data used to support the findings of this study are available from the corresponding author upon request.
